This article has been retracted.

# Magnetic Tile Surface Defect Detection Methodology Based on Self-Attention and Self-Supervised Learning

**DOI:** 10.1155/2022/3003810

**Published:** 2022-08-03

**Authors:** Xufeng Ling, Yapeng Wu, Rahman Ali, Huaizhong Zhu

**Affiliations:** ^1^Shanghai Normal University Tianhua College AI School, Shanghai, China; ^2^Key Laboratory of Intelligent Infrared Perception, Shanghai Institute of Technical Physics, Chinese Academy of Sciences, Shanghai, China; ^3^University of Peshawar, Peshawar 19120, Khyber Pakhtunkhwa, Pakistan

## Abstract

As the core component of permanent magnet motor, the magnetic tile defects seriously affect the quality of industrial motor. Automatic recognition of the surface defects of the magnetic tile is a difficult job since the patterns of the defects are complex and diverse. The existing defect recognition methods result in difficulty in practical application due to the complicated system structure and the low accuracy of the image segmentation and the target detection for the diversity of the defect patterns. A self-supervised learning (SSL) method, which benefits from its nonlinear feature extraction performance, is proposed in this study to improve the existing approaches. We proposed an efficient multihead self-attention method, which can automatically locate single or multiple defect areas of magnetic tile and extract features of the magnetic tile defects. We also designed an accurate full-connection classifier, which can accurately classify different defects of magnetic tile defects. A knowledge distillation process without labeling is proposed, which simplifies the self-supervised training process. The process of our method is as follows. A feature extraction model consists of standard vision transformer (ViT) backbone, which is trained by contrast learning without labeled dataset that is used to extract global and local features from the input magnetic tile images. Then, we use a full-connection neural network, which is trained by using labeled dataset to classify the known defect types. Finally, we combined the feature extraction model and defect classification model together to form a relatively simple integrated system. The public magnetic tile surface defect dataset, which holds 5 defect categories and 1 nondefect category, is used in the process of training, validating, and testing. We also use online data augmentation techs to increase training samples to make the model converge and achieve high classification accuracy. The experimental results show that the features extracted by the SSL method can get richer and more detailed features than the supervised learning model gets. The composite model reaches to a high testing accuracy of 98.3%, and gains relatively strong robustness and good generalization ability.

## 1. Introduction

The magnetic tile is an important component of the motor. Its quality will affect the performance of the motor, and the defects of the magnetic tile will lead to the decline of the performance of the motor, thus affecting the service life of the motor. If the defective magnetic tile is used in industrial robots or other industrial products, it will cause huge losses. We aim to develop a method to automatically detect the defects of the magnetic tiles in this study. The effect of traditional manual defect testing methods is easily influenced by individual experience and other subjective factors, which bring low consistency and efficiency. On the other hand, machine visual detection methods have the advantages of higher automation, good consistency, and noncontact measurement; therefore, they gradually become the mainstream methods of surface defect detection. Magnetic surface defect detection methods can be categorized into traditional image processing methods and deep learning methods [1, 2]. Zhu et al. [3] proposed a magnetic tile surface defect detection algorithm based on improved homomorphic filtering and the Canny algorithm to solve the problems of uneven illumination, low contrast, and grinding texture of magnetic tile images. The experimental results show that this method has a good effect on the surface defect detection of magnetic tile and high detection accuracy, and is suitable for many types of surface defects of magnetic tile. Zhang et al. [4] proposed a method to perform the visual detection of line defects on the surface of micromagnetic tile by using the adaptive static mask, masking the contour of micromagnetic tile, nonlinear anisotropic diffusion equation, and suppressing the surface texture of micromagnetic tile. The experimental results show that the algorithm can accurately extract the line defects in the surface image of magnetic tile, and the detection accuracy reaches to 94.6%. Ma et al. [5] proposed a method based on K-means clustering to segment the break defects of magnetic tile surface, conducted in-depth research on the selection of light source and K-means clustering algorithm, and used two algorithms to segment the image of magnetic tile surface. The experimental results show that the K-means clustering algorithm can correctly segment the break defects of the magnetic tile surface. The traditional image processing methods have the good systematic and strong logical characteristics, and achieve a good effect on many specific targets, but they are highly dependent on illumination, and show less robust and less ideal effects in practical applications.

Since 2012, the deep learning method has achieved continuous breakthroughs, VGG, GoogleNet, ResNet, and other networks that have been proposed by researchers, and the classification accuracy has been improved, especially the image visualization and semantic analysis algorithms [6, 7] continuously improves the deep learning technologies. Many defect detection frameworks using machine vision were applied in practice [8]. Convolutional neural network (CNN) has gradually become the leading method for recognition and detection tasks, and the deep learning method has also been deeply applied in magnetic tile detection. Xie et al. [9] proposed a defect segmentation and classification method based on U-Net, and they extracted the defect feature through the U-Net coding part, classified the defect using the feature, and then, output the segmented defect region through the decoding part. The experimental results show that the classification accuracy of this method is 98.9%, which meets the high-precision requirements of industrial production, and provides a new idea for the automation of magnetic tile surface quality detection. Guo et al. [10] proposed a defect detection algorithm based on the masked region with convolution network (Mask R-CNN), which mainly solved the problem that the traditional defect detection algorithm failed to accurately segment defects. Through the steps of image preprocessing, residual network ResNet-50, constructing feature pyramid network, regional proposal network (RPN), fully convolutional network for semantic segmentation (FCN), and fully connected layer for prediction, the algorithm realizes strong generalization ability and accurately segments the defects on tile images with complex surface texture, uneven illumination, and low contrast. Zhang et al. [11] proposed a deep convolutional generative adversarial network (GAN) using the Gaussian mixture model to generate magnetic tile images with defects, which solves the problems of difficult collection of magnetic tile defect samples, uneven number of different defect samples, single defect type, and so on. Based on GAN, the algorithm regards the input noise potential space of the generated image as the Gaussian mixture model, and can generate magnetic tile defect images with good quality and rich defect types. Zhang and Wang [12] proposed a magnetic tile surface quality recognition system based on the convolutional neural network. The magnetic tile target is segmented from the collected image and normalized to obtain the standard image. The multiscale ResNet-18 is used as the backbone network to design the recognition system; a novel in-class mix-up operation is designed to improve the generalization ability of the system to samples; and the recognition accuracy of the system can reach 97.9%. Aiming at the problems of unclear magnetic tile imaging, low contrast, complex texture background, and many types of defects, Hu et al. [13] divided the types of magnetic tile surface defects into three categories and designed defect extraction methods, respectively, according to the different characteristics of the three types of surface defects. The experimental results show that this method can accurately and quickly extract the defect region on the surface of magnetic tile, and the detection accuracy is 93.5%. Li et al. [14] proposed a magnetic ring surface defect detection method based on the masked image. The magnetic ring surface defects are divided into two categories. According to the imaging characteristics of the two types of surface defects and their relationship with the background, the corresponding defect extraction methods are designed to use mask technology. Finally, many online experiments are carried out on samples with different illumination, specifications, defect types, and sizes. The experimental results show that this method has strong robustness, which can accurately and quickly extract the defects in each region of the magnetic ring surface image, and the detection accuracy reaches 95.3%.

Compared with traditional machine vision methods, the main advantage of deep learning methods is that they can automatically extract latent features without doing any manual feature engineering jobs like traditional methods, and have better robustness and adaptability in practical applications [15–17]. At present, the deep learning methods of magnetic tile image defect detection are all supervised learning methods. Nowadays, the supervised learning is the most common machine learning method. Given the dataset labeled manually in advance, the machine can learn to map the input data to the labeled target. Supervised learning has two disadvantages: first, it needs enough labeled training datasets including images, text, and voice, which mostly needs to be built manually. The data annotation process is a time-consuming and expensive process. In some areas, such as the medical field, obtaining a big labeled dataset is a challenging job. Second, data annotation will lead to information loss. For example, an image contains very rich information, including background information and secondary target information in addition to labeling objects. A single training task only extracts the information related to the training target in the image and ignores other valuable information. To solve the shortcomings of the supervised learning method, a single-stage defect recognition method, which integrates defect detection and defect classification together of magnetic tile, is proposed in this study, a similar job what our team did in another research [18]. This method uses a deep neural network model based on the self-supervised learning methodology.

The key contributions of the proposed method include the following:

- An efficient multihead self-attention mechanism is proposed, which automatically locates single or multiple defect areas of magnetic tile and extracts features of the magnetic tile defects
- The design of an accurate full-connection classifier can accurately classify different defects of magnetic tile defects.
- A knowledge distillation process without labeling is proposed, which simplifies the self-supervised training process.
- A flexible backbone network selection methodology is proposed, which can select suitable networks such as ViT and ResNet without changing the whole network structure.

In this study, the self-supervised learning network is used to train the encoder to do the feature extraction job. The backbone network is ViT. We make full use of the existing pretrained models to evaluate the classification effects of the target task. If there exists any pretrained model, which meets the requirements, then it can be directly used; otherwise, we use the self-supervised learning method to fine-tune the pretrained model. We also train a fully connected linear classifier MLP to do the classification task.

The rest of the study is structured as follows.  Section 2 describes in the proposed research methodology.  Section 3 realizes the proposed methodology by performing experiments and analyzing the results, and Section 4 concludes the research work did in this study.

## 2. Proposed Research Methodology

Since 2020, the self-supervised learning has increasingly attracted people's attention and become the most promising development direction at present [19]. Self-supervised learning is a supervised learning without human participation. It is not unsupervised learning [20–22]. With the exquisite design, it realizes self-supervised learning from the relationship of training data. Labels are generated from input data and are usually generated by the heuristic algorithm.

At present, the self-supervised learning of machine vision can be divided into two types: generative self-supervised learning and discriminant self-supervised learning [20, 23]. The main methods of generative self-supervised learning are VAE and GAN. The main idea is to train a model with the goal of learning the internal relationship of image pixels and then mask a part of the image, requiring the model to reconstruct or restore the obscured part of the image. This type of task is relatively difficult, because the model can reconstruct the image at the pixel level only when it has rich detailed information. The typical method of discriminant self-supervised learning is contrastive learning. Contrastive learning is to train a feature extraction model by automatically constructing similar and dissimilar instances. Through this model, similar instances are close in the projection of feature space, while dissimilar instances are far away in the projection space. The key points are how to construct similar and dissimilar instances, how to construct a model structure, and how to prevent model collapse. In general, compared with generative self-supervised learning, contrastive learning is less difficult.

At present, there are many kinds of self-supervised learning methods [24, 25] that can be roughly divided into two categories. The first one is generic self-supervised learning, such as scene occlusion removal, depth estimation, optical flow estimation, and image correlation point matching. The second one is discriminant self-supervised learning with the typical methods, such as solving jigsaw puzzles, motion propagation, rotation prediction, MoCo, and SimSam. The method in this study mainly refers to the method of Caron et al. [24] and belongs to the second category.

### 2.1. Workflow of the Proposed Methodology

To solve a coming downstream task such as an image classification task, the first step is data preparation, and an appropriate dataset for the task is to be carefully chosen. The second step is the model collection, and each modal *M*_1_, *M*_2_,…, *M*_*n*_ in the model zoo is taken out. The third step is KNN evaluation [26], and each existing pretrained model is evaluated by the KNN method to find whether there exists a model whose KNN classification accuracy exceeds 80%. If there is no pretrained model that meets the requirement, then we must do the step 4, using the self-supervised learning method to retrain a new model to improve its feature extraction performance, and go to the fifth step; on the contrary, if there exists model *M*_*K*_ that meets the requirement, then we do not need to retrain a new model; we can then do the fifth step; and the pretrained model *M*_*K*_, which has relatively good feature extraction performance, will be fine-tuned to improve its classification ability. The fine-tuning job is to train an MLP (a fully connected linear classifier) attached to the feature extraction model, to complete the downstream classification. The process of the method is shown in Figure 1. The sixth step is result analysis to do research on the method.

### 2.2. The Backbone Network (ViT)

The backbone network of contrastive learning in this study is the ViT [27]. Compared with the convolutional neural network CNN, the attention-based ViT method can achieve better results in image recognition, mainly because ViT can realize self-supervised learning. The model design of ViT in this study is basically consistent with the transformer architecture in the initial natural language processing [28]. This has three very significant advantages: first, the model setting is simple. Second, it is similar to transformer and has good scalability. Third, it is out of the box with efficient implementation. The architecture of ViT model is mainly composed of five parts: image patch segmentation, image patch embedding, position embedding, sequence of self-attention modules, and a fully connected layer MLP that acts as a classification header. First, the input image is divided into *N* × *N* image patches, and each image patch is embedded into a vector (called image block embedding) through a fully connected network. Each image patch can be represented as a word, and the input image can be represented as a *N* × *N* word sequence. Then, we add an additional learnable token (called CLS), which may synthesize the information of the whole sequence at the head of the sequence. The task of image classification is transformed into the semantic recognition task. Next, we design the ViT network with sequence length *L*, dimension *D*, and *K* attention modules cascaded. Finally, there is a full-connection layer MLP, which realizes the classification function as a downstream task. The network structure is shown in Figure 2.

In this study, the input image size is 224 × 224 pixels; the patch is 16 × 16 pixels; and the image is split into 14 × 14 patches. There are 12 multi-self-attention head blocks cascaded to form the backbone network, and the main job of the backbone network is feature extraction. Each block holds 12 heads; the embedding dimension is 768; and the sequence length is 197. The MLP is for the downstream classification task.

### 2.3. Contrast Learning

The contrastive learning network consists of the student network and the teacher network. The student network and the teacher network are two ViT networks with the same structure but different parameters. For the input image *x*, the random image change transforms the image *x* into *X*1 and *X*2, respectively. *X*1 is input to the student network, and *X*2 is input to the teacher network. The *k*-dimensional feature outputs from the student network are normalized by softmax (taking the temperature parameter *t* as the denominator in the feature dimension) to obtain the probability distribution *P*1. The probability of the output of the teacher network is *P*2. To avoid the network collapse in the process, two skills, namely, averaging and sharpening, are adopted. Cross entropy is used to calculate the similarity between the student network output and the teacher network output. Because it is the input of different transformations of the same image, the error of the two network output distributions *P*1 and *P*2 is required to be small enough. The error loss is gradient backpropagated to the student network, while the teacher network does not. The update of the teacher network parameters is completed by an exponential moving average of the student network parameters. The model structure is shown in Figure 3.

### 2.4. Implementation Process

The student network *g*_*θ*_*s*__ (the parameter is  *θ*_*s*_) needs to be trained to get the same results as the output of the given teacher network *g*_*θ*_*t*__ (the parameter *θ*_*t*_). Thus, for an input image **X**, the **K**-dimensional output probability distribution of the two networks is denoted as *P*_*s*_ and *P*_*t*_. The probability distribution **P** can be obtained by softmax normalization of the network *G* output, that is, formula (1)as follows:

(1) $$\begin{array}{c} P_{s}{\left(x\right)}^{i}=\frac{\left(\exp\left(g_{\theta_{s}}{\left(x\right)}^{i}/\tau_{s}\right.\right)}{\sum_{k=1}^{K}\exp\left(g_{\theta_{s}}{\left(x\right)}^{k}/\tau_{s}\right)}. \end{array}$$

Here, *τ*_*s*_ is a temperature parameter that controls the steepness of the output distribution. The smaller the value of *τ*_*s*_, the steeper it is; and the larger its value, the smoother it is. Given teacher network on the premise of *g*_*θ*_*t*__, we match the output distribution of the two networks by minimizing the cross entropy.

(2) $$\begin{array}{c} \text{min}H\left(P_{t}\left(x\right),P_{s}\left(x\right)\right). \end{array}$$

Here, *H*(*a*, *b*)=−*a*log*b*. Next, we describe formula (2) in detail. First, we intercept and deform the input image, construct different views, and form the view set *v*. This collection includes 2 global views (*x*_*g*1_, *x*_*g*2_) and 8 local views (*x*_*l*1_, *x*_*l*2_,…, *x*_*l*8_). The global view is only available to the teacher network; all views are available to the student network. The local-global similarity is formed in this way, and the training process is to minimize the loss as described in formula (3)as follows:

(3) $$\begin{array}{c} \text{loss}=\text{min}\sum_{x\in x_{1}^{g},x_{2}^{g}}\sum_{x^{\prime }\in Vx^{\prime }\neq x}\left.H\left(P_{t}\left(x\right)\right.,P_{s}\left(x^{\prime }\right)\right). \end{array}$$

The image resolution is set to 224 × 224, and the size of the global view is set to (0.4–1) to cover a large area of the input image, while the size of the local view is set to (0.15–0.4) to cover only a small area of the input image. The parameters of the network can be trained out by minimizing the formula (3) of random gradient descent *θ*_*s*_.

### 2.5. Candidate Pretrained Model Selection

The pretrained model has two very valuable characteristics: first, the features extracted by the self-supervised ViT method can have image segmentation ability, including scene layout and object boundary. This information can be obtained by extracting the self-attention features of the last layer. Second, the features extracted by self-supervised DINO-ViT do not need any fine-tuning, linear classifier, or data enhancement. Only the most basic KNN method can achieve a good classification effect, and the top-1 accuracy on ImageNet [29] can reach 78.3%. This study proposes a self-supervised learning model based on the combination of contrastive learning and self-attention mechanism for magnetic tile recognition.

There are a series of open-source pretrained models based on ImageNet on GitHub. Some models are listed in Table 1 [29]. These models have good performance in ImageNet and can be directly used or after training and tuning. Table 1 contains self-supervised feature extraction models with different parameters, in which “Layers” refers to the layers of transformer; “Dimension” refers to the working dimension of transformer; “Number of heads” refers to the number of heads with attention, similar to the number of convolution kernels in CNN; “Token number” refers to the length of embedded code; and “Parameter quantity” refers to the total parameters of the model, excluding the parameters of the MLP full-connection layer.

Each existing pretrained model is validated to find out whether it can meet the requirement. For ViT-S/8 & ViT-6/8, 8 stands for small image patch with 8^*∗*^8 pixels, with the input image 224^*∗*^244; it has longer patch sequence of 785 and has 4 times heavier computation than ViT-S/16 and ViT-B/16, respectively; and meanwhile, the classification accuracy is improved only by 1–2%. Finally, we choose ViT-B/16 to do extensive experiments, so it has the balance between performance and computation.

## 3. Experimental Results and Analysis

The SSL-ViT model proposed in this study is trained, verified, and tested on the open data of magnetic tile. The experiment is completed on a server configured with four RTX 2080Ti GPUs. The server operating system is CentOS 7.6 and memory is 128G. The program is implemented in Python language and is completed on the Python 1.60 deep learning platform. The specific experimental work includes selection of magnetic tile image dataset, image data preprocessing, model training, model optimization, model test, comparative experiment, and so on.

### 3.1. Data Preparation

The experimental dataset in this study is the magnetic tile surface defect dataset. The dataset was collected by Huang from the Institute of Automation, Chinese Academy of Sciences, in order to detect and identify five defects in industrial magnetic tile. The defects in the dataset are blowhole, crack, break, fray, and unevenness. Each defect has dozens to hundreds of gray images, and the size of each gray image is also inconsistent. We randomly divided the dataset into training set, verification set, and test set, with a ratio of 8 : 1 : 1.

The dataset is shown in Table 2. It can be seen from the table that a large number of pieces, i.e., 952, are without defects. The fray category of defect data is less, and other categories are relatively balanced. The number of data samples is small; the large dataset needs to be enhanced through data enhancement; and then, we can reduce the dependence of the model on irrelevant attributes, and improve the robustness and generalization ability of the model. An online data augment method is used to increase the samples; each sample of the dataset is translated, resized, flopped, and stretched to produce more samples. Since the experimental platform is PyTorch, many methods in torchvision package such as RandomResizedCrop, RandomHorizontalFlip, RandomRotation, and RandomAffine are used to achieve online data augmentation operation.

### 3.2. Retraining of Pertained Model

The existing pretrained model is trained on ImageNet and has good image feature extraction functions. Because ImageNet images are mainly images in nature, the pretrained model has a strong ability to extract the characteristics of natural images. As an industrial product, the visual characteristics of magnetic tile are significantly different from natural objects, and the direct use of the pretrained model may result in poor effects. However, this does not mean that the pretrained model is worthless, and the basic visual feature extraction function is very valuable. We import the pretrained model and then train it with the magnetic tile dataset, so that the model can extract the magnetic tile features well.

We can judge a pretrained model as whether it can do a good feature extraction job for a certain dataset such as the magnetic tile dataset by simply using KNN (K-nearest neighbor, an automatic classification method) validation [11]. Experiments show that if the classification accuracy of KNN validation of a pretrained model on a certain dataset is above 80%, the feature extraction effect of the pretrained model is good, and the next job is to fine-tune the model to achieve better downstream classification task. If the KNN validation gets a low classification accuracy score, the pretrained model cannot extract features well from the task of the certain dataset, and the next job is to choose another pretrained model or retrain a new model to improve its feature extraction ability. In this study, the KNN classification accuracy of the pretrained model is 67.35%, which cannot meet the requirements; therefore, the pretrained model cannot be used and need to be retrained. The pretrained model is retrained over the magnetic tile dataset to optimize its feature extraction ability. The training epoch is set to 200. The optimizer is set as ADM, and the learn rate is set as the cosine optimization scheme. The training loss and learn rate are shown in Figure 4.

During the retraining of the pretrained model with the magnetic tile data, the training error change curve is shown in Figure 4(a). With the increase in epoch times, the training error decreases. When the epoch reached 100, the training error would basically converge. When the epoch reached 200, the training error would converge to about 3.9. Figure 4(b) shows the change curve of learning rate. The warm-up linearly increases in the first 30 cycles (this is a skill to improve training efficiency) and then gradually decreases.

### 3.3. KNN Estimation and MLP

When the training period exceeds 100, the decline speed of training error will slow down; when the training period exceeds 150, the training error will tend to converge; then, the retraining of the pretrained model is basically completed; and the feature extraction network is optimized. Next, we use KNN to evaluate the feature extraction ability of the model. The results are shown in Table 3.

Because the number of samples in the dataset is relatively small, when the *N* increases, the classification accuracy of KNN decreases. Generally, we take *N* = 10 as the reference basis, and the classification accuracy reaches 94.7%. Therefore, we have reasons to believe that the trained model has a good ability of magnetic tile feature extraction.

Next, we train a fully connected network MLP to classify features, that is, applying the linear classifier training to realize the classification function. This is a downstream task and a training process of supervised learning. The ratio of training set, verification set, and test set is 8 : 1 : 1; epoch is set to 100; and the training process is shown in Figure 5. We can see that the change curve of training error and verification error is shown in Figure 5(a). The loss value of training set and test set gradually decreases with the increase in epoch. When the epoch value is greater than 40, the training error hardly decreases; the verification error also changes very little; and the change curves of classification accuracy of training set and the verification set are shown in Figure 5(b). With the increase in epoch times, the accuracy of training set and verification set increases. Finally, the accuracy of verification set is 98.25%.

We train a feature extraction network to realize image feature extraction through self-supervised learning and then learn a linear classifier through a supervised learning method to complete the downstream classification task. This hybrid model of self-supervised learning combined with supervised learning not only achieves a good classification effect, but also improves the universality of the model, reducing the threshold of practical application, and has a broad application prospect.

### 3.4. Comparative Test and Analysis

We conducted a comparative experiment and compared it with the Swin-ViT, ViT, and ResNet-50 using supervised learning. We found that if we do not do region extraction and other work, and directly use the supervised learning Swin-ViT, T2T-ViT, and ResNet50 networks to classify magnetic tiles, the classification accuracy of all the supervised methods does not exceed 80.0%, as shown in Table 4. Because the defects of the magnetic tile are open and have no fixed mode. In this case, if the defect region is not extracted in advance, the traditional supervised learning method is difficult to accurately extract features of the magnetic tile, and it is difficult to achieve high classification accuracy.

### 3.5. Attention Map Analysis

The model has multiple attention heads. The experimental model in this study has six attention heads, and each attention head focuses on different attention regions. We note that the attention area of each attention head is very similar to human visual characteristics. The areas that the attention heads pay attention to are those with very rich information. Further observation and research show that the defect areas will be noticed by one or more attention heads. This is the advantage of self-supervised learning. It is not affected by label data, and the learned features are very comprehensive. Self-supervised learning has a better effect on open tasks than on closed tasks. We carefully analyzed the model feature extraction and attention map, which is shown in Figure 6.

In Figure 6, the left side is the attention map and the right side is the original image.  Figure 6(a) is a blowhole defect; Figure 6(b) is a crack defect; Figure 6(c) is a break defect; Figure 6(d) is a fray defect; and Figure 6(e) is an unevenness defect. The feature extraction method of the self-supervised model is richer and more detailed, which can automatically pay attention to the location of defect attention, and find the abnormal region location. For complex industrial vision, using a self-supervised method can have a good effect.

The self-attention maps contain information about image segmentation. Different attention heads can process different semantic regions of an image, even if they are occluded. ViT of supervised learning cannot deal with messy objects well, both qualitatively and quantitatively. On the contrary, self-supervised ViT can deal with these objects. Even if the scene is very complex, the defect area of the image can be segmented from the complex nondefect background by multiple attention heads. We believe that the SLL method pays attention to the abnormal areas of the image and separates the abnormal region from the normal region. But sometimes, abnormal areas are nondefect area, and in this case, we need a downstream MLP to do further nonlinear classification to solve this problem.

## 4. Conclusions

To solve the difficult task of magnetic tile defect detection of industrial product quality control job, we use self-supervised learning method for feature extraction and combined supervised learning method for the downstream classification task, to detect the defects of the magnetic tile. This method will be able to undertake a single-stage magnetic tile defect detection. The open-source magnetic tile surface defect dataset, which contains five defect categories, is used in this research. The experimental results show that the self-supervised learning method has unique advantages in feature extraction. First, multiple self-attention heads can automatically locate different defect locations. Second, the model holds image segmentation information of complex scenes. Third, the model has strong feature extraction and generalization ability. The above characteristics show that the self-supervised method can extract global semantic features and local detail features. The model uses the fully connected network to complete various downstream classification tasks. Since the above method is flexible and convenient, it holds practical application value for many industrial product quality inspections. In addition, the self-supervised learning model has a good application prospect in the field of industrial images. The dataset we use to train and test our method in this study is relatively not big enough, and we need to collect more samples of magnetic tile defects to develop a larger dataset to train and test our method in the next study. The future work is to test the self-supervised learning model in multiple industrial scenes, develop a self-supervised learning feature extraction model with excellent generalization, develop a lightweight model that can be applied in smart manufacturing, and also find out whether the industrial conditions like temperature and humidity affect the results of this study. A practical magnetic tile defect detection system will be widely used in smart manufacturing and bring huge economic benefits.

## Figures and Tables

**Figure 1:** Workflow of the proposed method.

**Figure 2:** Network structure of ViT, and MSA denotes multi-self-attention head block.

**Figure 3:** Architectural design of self-supervised DINO model; SG indicates no reverse gradient propagation; and EMA indicates exponential moving mean update.

**Figure 4:** Schematic diagram of training loss and learning rate, and the pretrained model is ViT-B/16.

**Figure 5:** Linear classification training, testing loss, testing accuracy, and the pretrained model are ViT-B/16.

**Figure 6:** Original images of various defects and self-attention images. Different colors denote different attention scale; yellow denotes high attention; bright green denotes common attention; and dark green denotes low attention. (a) Blow hole. (b) Break. (c) Crack. (d) Fray. (e) Uneven.

**Table 1:** List of parameters of pretrained model.

Model	Layers	Dimension	Heads	Tokens	Parameters (M)
ResNet-50	—	2048	—	—	23
ViT-S/16	12	384	6	197	21
ViT-S/8	12	384	6	785	21
ViT-B/16	12	768	12	197	85
ViT-B/8	12	768	12	785	85

**Table 2:** Magnetic tile defect dataset details.

Category	Blowhole	Crack	Break	Fray	Uneven	Free
Number	115	114	85	32	103	952

**Table 3:** Estimation of KNN classification accuracy, N means, and N neighbors.

N	5 (%)	10 (%)	20 (%)	30 (%)

Classification accuracy	96.9	94.7	86.5	81.2

**Table 4:** **C**omparison of SLL method with other supervised methods.

*N* Nearest-neighbor method	RestNet-50	ViT-base	Swin-ViT-base	SSL method
Top-1 accuracy	63.0%	67.7%	78.5%	98.3%
Epoch	200	200	200	200

## Data Availability

Data can be provided on the request.
